# A Computational Framework to Study the Effect of Acupuncture on Obesity by Integrating Multiple Levels of Data

**DOI:** 10.1155/2020/8513860

**Published:** 2020-10-16

**Authors:** Huihui Liu, Mingjun Liu, Yingbo Jiao, Le Wei, Xiaochen Liu, Dandan Li, Xiaolin Zhang, Minghui Yan, Jinming Chen

**Affiliations:** ^1^Chifeng Municipal Hospital, Chifeng, China; ^2^Changchun University of Chinese Medicine, School of Acupuncture-Moxibustion and Tuin, Changchun, China; ^3^Chifeng Education Center for CPC Member, Chifeng, China; ^4^Chifeng Cancer Hospital, Chifeng, China

## Abstract

In this study, we evaluated the efficacy of acupuncture in the treatment of obesity by a computational framework integrating randomized controlled trials published in China and abroad. Specifically, clinical trial documents published on CNKI, VIP, Wanfang, PubMed, Embase, and the Cochrane Library from 2007-2017 were downloaded and analyzed using Stata 15.1 system. As a result, a total of 13 articles were imported and 1052 patients were included. The analyses showed that the overall effect of an acupuncture group and a control group was not significant with *P* > 0.01. However, the curative effect of the acupuncture group was better than that of the diet and exercise instruction group with *P* < 0.01; the curative effect of the acupuncture group was better than that of the oral Chinese and western medicine group with *P* < 0.01. In conclusion, acupuncture as a complementary alternative therapy is recommended for the treatment of obesity.

## 1. Introduction

Obesity mainly refers to the exclusion of excessive systemic fat accumulation caused by hereditary, metabolic, traumatic, or other diseases. A survey by JAMA shows that 2/3 of people in the United States are overweight or obese [1]. Another survey report shows that Americans pay $147 billion a year for obesity-related diseases and the number of obese people in China is also increasing. A survey by the Chinese Center for Disease Control and Prevention showed that in 2003 alone, the direct economic burden caused by obesity in four chronic diseases (hypertension, coronary heart disease, diabetes, and stroke) was as high as 2.01 billion Chinese yuan, accounting for 25.5% of the total direct disease burden of the four diseases [2, 3]. With the continuous progress of people's understanding of medicine, some complementary alternative medical methods have gradually become the first choice for people who lose weight. In 1998, the consensus meeting of the National Institutes of Health issued a statement about the promising results of acupuncture in the treatment of some diseases such as obesity [4].

The purpose of this study was to eliminate the confounding factors of intervention measures such as electroacupuncture, ear acupuncture, and auricular point pressing, to conduct a meta-analysis on the results of clinical high-quality randomized controlled trial (RCT) published in 2007-2017 on acupuncture treatment of obesity, and to evaluate and summarize the weight loss effect of acupuncture on obesity to provide evidence for clinical treatment.

## 2. Method

### 2.1. Retrieval Strategy

The search scope of this study includes Chinese databases from January 2007 to October 2017: China knowledge Network, Wanfang, VIP, and Baidu academic databases, and English databases: PubMed, Embase, and Cochrane Library. The Chinese database search strategy is as follows: obesity or obesity or overweight or weight loss or weight loss or weight control or slim and acupuncture or acupuncture or embedding therapy or electroacupuncture or ear acupuncture or degree catgut embedding or auricular point pressing or moxibustion or traditional Chinese medicine acupuncture or body acupuncture or manual acupuncture or clinical trial or clinical study or clinical efficacy or effectiveness; the English database determines the search strategy through MeSH and textwords: simple obesity OR obesity obese OR overweight OR weight loss OR weight Control OR weight reduction OR overweight OR overeat AND acupuncture OR electro acupuncture OR auricular acupuncture OR acupressure OR acupoint OR moxibustion AND random AND controlled clinical trial AND trial. At the same time, the conference papers and academic reports related to obesity were searched to reduce the risk of publication deviation.

### 2.2. Inclusion Criteria

1. Study design: all clinical randomized controlled trials of acupuncture in the treatment of obesity do not limit the use of blind methods, but the principle of random distribution must be adopted
2. Intervention: the observation group was treated with manual acupuncture, in which acupuncture manipulation, location, and time were not limited, while the control group was treated with nontraditional manual acupuncture
3. Subjects: subjects are selected in accordance with the clinical diagnostic criteria of “obesity” [5–7]
4. Outcome indicator: the outcome indicators are as follows: body mass (BM) and body mass index (BMI)
5. All the subjects were from 13 to 69 years old, with a balanced male-to-female ratio, no restrictions on race, and no restrictions on the course of disease between the gender observation group and the control group
6. Provide full text and complete data

### 2.3. Exclusion Criteria

1. The exclusion criteria are obesity syndrome patients, pregnant women, and abdominal obesity
2. The observation group was treated with acupuncture, electroacupuncture, ear acupuncture, auricular point pressing, acupoint catgut embedding, and other treatments
3. The control group was treated with manual acupuncture, but the acupuncture method, location, and time were different
4. All the subjects were 13 years old and over 69 years old, and the sex of the observation group and the control group was single male or female

### 2.4. Evaluation Standard of Curative Effect

Refer to the standard of efficacy of obesity discussed at the first national conference on the treatment of obesity by Integrated traditional Chinese and Western Medicine in 1987 [5]. Recovery is defined asweight loss > 80%and body mass index (BMI) 25-28. Significant effect is defined as weight loss 30%, Mel 70%, and body mass index (BMI) drop > 4. Effective means weight loss 25%, Mel 30%, and body mass index (BMI) drop ≥ 2. Ineffective means weight loss < 25% and body mass index (BMI) > 30 kg/m^2^.

### 2.5. Data Extraction and Document Quality Evaluation

Two independent reviewers (LXC, LDD) searched the literature, including title, abstract, and full text, respectively, and consulted a third researcher to resolve differences on controversial studies. The information of the included literature was extracted, including first author, year of publication, country, research design, sample size, treatment measures of the observation group and control group, course of treatment, results, implementation of blind method, outcome index, course of treatment, and inclusion criteria. The systematic review manual (version 5.3.0) provided by the Cochrane collaboration Network was used to evaluate the bias risk of the included studies, including (1) the generation of random allocation scheme; (2) covert grouping; (3) blind method for patients and doctors; (4) blind method for outcome evaluation; (5) incomplete result data; (6) selective result report; and (7) other biases. Each item is rated as “yes,” “no,” or “unclear”; “yes” indicates a high risk of bias, “no” indicates a low risk of bias, and “unclear” indicates that the risk of bias is uncertain or unknown. When there are differences in the results of the assessment, it will be discussed and resolved by two commentators (JYB, WL).

### 2.6. Data Analysis

In this experiment, RevMan 5.3 software is used to make a flow chart and PRISMA scale. Stata 15.1 software was used for meta-analysis. The weighted average difference (WMD) and its 95% CI confidence interval are used as the statistical measures of effect analysis; *Q* test and *I*^2^ are used to evaluate heterogeneity; if *I*^2^ ≥ 50% or *P* < 0.1, the results of each study may have heterogeneity; a random effects model is used for combined analysis [7, 8]; Galbraith diagram is drawn to detect the sources of heterogeneity; and Egger's test is used to detect the existence of publication bias [9, 10]. Subgroup analysis was used to compare the efficacy of different factors in each trial.

## 3. Result

### 3.1. Description of the Inclusion Trial

In this study, a total of 413 articles were obtained through manual retrieval, and 42 were retrieved through conference papers and academic reports. Through the screening of titles and abstracts, 164 articles were deleted and the remaining 291 articles were left. The whole article was read and 46 articles published repeatedly were deleted, 65 were nonclinical randomized controlled trials, 21 were experimental studies, 3 were health investigation reports, 68 were acupuncture and moxibustion combined with other therapies in the observation group, and 88 articles were left. In further qualitative analysis, 59 studies that were not in accordance with the inclusion trial were deleted, of which 4 were female; 43 were included in the observation group with manual acupuncture combined with electroacupuncture and ear acupuncture; and 12 were included in the study with three groups of controls. 29 studies were included in the preliminary systematic review, and 7 articles that did not mention random allocation methods and 9 articles with insufficient data were excluded according to the quality criteria of the included literature. Finally, 13 relatively high-quality RCT were included in the meta-analysis, as shown in Figure 1.

This study included 13 trials and 1052 subjects, published from 2007 to 2017, aged from 13 to 69 years old; regardless of the course of disease, the course of treatment was between 4 and 12 weeks, and the time of single acupuncture was 30 minutes.

### 3.2. Bias Risk of Inclusion in the Study

According to the methodological quality assessment item 1 provided by the Cochrane Collaboration Network, the generation of random allocation scheme is as follows: 2 covert grouping; 3 blind method for patients and doctors; 4 blind method for outcome evaluation; 5 incomplete result data; and 6 selective result report; 7 other biases were included in the literature quality evaluation; 13 trials described random assignment; and 3 [11–13] trials described the blind method and were single blind. Zero trials described the withdrawal of cases, and 0 trials were followed up. Through the evaluation, we can know that the quality of the 13 trials is average, and the random allocation scheme is low risk, but whether to implement blind method for patients and doctors and blind method for result evaluation is high risk, and covert grouping is also high risk. The summary results are shown in Figure 2.

### 3.3. The Meta-Analyses of the Effect of Acupuncture on Body Weight and Body Mass Index of Obesity

The results of meta-analysis of 13 trials showed that the effect of acupuncture on improving body weight and body mass index of obesity was not significant compared with the control group [11–23]: WMD = −3.07, 95%CI = −7.02~0.88, *P* = 0.127; heterogeneity was higher than that of the control group. 99.4% of WMD = −3.07, 95%CI = −7.02~0.88, *P* = 0.127, and heterogeneity was higher than that of the control group (see Figure 3(b)).

### 3.4. Galbraith Heterogeneity and Egger's Test

The results of Galbraith heterogeneity test are as follows: there were two tests in weight test, and the scatter map was obviously distributed beyond the two regression lines, which was the main source of heterogeneity (see Figure 4(a)) [15, 20]. Body mass index test showed that the scatter plot was obviously distributed outside the two regression lines in three tests, which was the main source of heterogeneity, as shown in Figure 4(b) [15, 18, 23].

The results of weight Egger's test are as follows: *P* = 0.23 and *P* > 0.1, and no significant publication bias was detected. The body mass index Egger's test results are as follows: *P* = 0.13 and *P* > 0.1, and no obvious publication bias was detected.

### 3.5. Subgroup Analyses

The results of subgroup analysis are as follows: the results of subgroup analysis of different intervention measures in the control group: group 1: WMD 1.27 95% CI (-4.70, 7.23), *P* = 0.68; WMD 0.58 95% CI (-2.37, 3.52), *P* = 0.70; group 2: WMD -2.06 95% CI (-4.38, 0.26), *P* = 0.08; WMD -1.15 95% CI (-2.33, 0.04), *P* = 0.06; group 3: WMD 3.40 95% CI (-4.20, -2.60), *P* < 0.01; WMD -1.37 95% CI (-1.79, -0.95), *P* < 0.01; and group 4: WMD-14.54 95% CI (-15.55, -13.53), *P* < 0.01; WMD -0.75 95% CI (-0.94, -0.56), *P* < 0.01. The combined effect values of each subgroup showed that the curative effect of acupuncture was better than that of sham acupuncture and diet and exercise guidance, as shown in Figures 5(a) and 5(b).

## 4. Discussion

### 4.1. Methodological Quality of Inclusion in the Study

This study found that there were methodological quality problems in most clinical trials of acupuncture treatment of obesity: the blind method was implemented in 3 trials. There are high risks in 13 trials in three aspects: hidden grouping, blind method for patients and doctors, and blind method for result evaluation, but these risks are related to trial interventions. Acupuncture treatment requires manual operation, which has special limitations compared with simple medication. Through the summary, we can know that sham acupuncture can well avoid a variety of risks of experimental research, and it is suggested that more sham acupuncture control group trials should be carried out in the future, so as to clarify the efficacy of acupuncture in the treatment of obesity.

### 4.2. Efficacy and Safety

The results of meta-analysis showed that acupuncture had no significant effect on body weight and body mass index (BMI) of obesity, but acupuncture had a more significant effect on patients with a course of treatment of less than 8 weeks. At the same time, the effect of acupuncture was better than that of sham acupuncture and diet and exercise guidance. However, because the number of trials guided by sham acupuncture and diet and exercise in the control group is less and the results are not robust, more clinical randomized controlled trials are needed in the future to ensure the therapeutic advantage of acupuncture. The heterogeneity of 13 trials was relatively high, and we used the random effects model to deal with the heterogeneity, but it did not decrease. The heterogeneity of Galbraith diagram was tested, and the sources of heterogeneity mainly included 4 trials [15, 18, 20, 23]. Through the further interpretation of the four trials, we found that the source of heterogeneity may be related to the intervention measures in the control group, which are mainly drugs in the control group. The second source of heterogeneity may be that the *R* value of each index is different from that of the trial *R* value which does not give the difference in curative effect, and the third reason may be that the patients participating in these trials are evenly distributed between the ages of 18 and 50 years old. The fourth reason may be related to the uneven distribution of the short or long course of disease in the patients involved in the trial.

## 5. Conclusion

In this study, the randomized controlled trials of acupuncture in the treatment of obesity were analyzed and summarized. It can be seen that the effect of acupuncture in the treatment of obesity is positive, and it is a recommended green clinical alternative therapy.

## Figures and Tables

**Figure 1:** Flow chart of literature retrieval and screening.

**Figure 2:** Methodological quality evaluation form.

**Figure 3:** (a) Forest map of body weight. (b) Body mass index forest map.

**Figure 4:** (a) Weight test chart of Galbraith. (b) Detection of body mass index of Galbraith.

**Figure 5:** (a) Forest map of the effect of different intervention measures on body weight. (b) Forest map of the effect of different intervention measures on body mass index.

## Data Availability

The analyzed data sets generated during the present study are available from the corresponding author on reasonable request.
